RETRACTED

# The Anti-Inflammatory Effects of Shinbaro3 Is Mediated by Downregulation of the TLR4 Signalling Pathway in LPS-Stimulated RAW 264.7 Macrophages

**DOI:** 10.1155/2018/4514329

**Published:** 2018-04-05

**Authors:** Hwa-Jin Chung, Wonil Koh, Won Kyung Kim, Joon-Shik Shin, Jinho Lee, Sang Kook Lee, In-Hyuk Ha

**Affiliations:** ^1^Jaseng Spine and Joint Research Institute, Jaseng Medical Foundation, Seoul 135-896, Republic of Korea; ^2^College of Pharmacy, Natural Products Research Institute, Seoul National University, Seoul 151-742, Republic of Korea

## Abstract

Shinbaro3, a formulation derived from the hydrolysed roots of *Harpagophytum procumbens* var. *sublobatum* (Engl.) Stapf, has been clinically used in the pharamacopuncture treatment of arthritis in Korea. In the present study, Shinbaro3 inhibited NO generation in LPS-induced RAW 264.7 cells in a dose-dependent manner. Shinbaro3 also downregulated the mRNA and protein expression of inflammatory mediators in a dose-dependent manner. Three mechanisms explaining the effects of Shinbaro3 in RAW 264.7 cells were identified as follows: (1) inhibition of the extracellular signal-regulated kinase 1 and 2 (ERK1/2), stress-activated protein kinase (SAPK)/c-Jun N-terminal protein kinase (JNK), and p38 mitogen-activated protein kinase (MAPK) pathways; (2) suppression of I*κ*B kinase-*α*/*β* (IKK-*α*/*β*) phosphorylation and nuclear factor-kappa B (NF-*κ*B) subunits in the NF-*κ*B pathway, which are involved in MyD88-dependent signalling; and (3) downregulation of IFN-*β* mRNA expression via inhibition of interferon regulatory factor 3 (IRF3) and Janus-activated kinase 1 (JAK1)/signal transducer and activator of transcription 1 (STAT1) phosphorylation, which is involved in TRIF-dependent signalling. Shinbaro3 exerted anti-inflammatory effects in LPS-stimulated RAW 264.7 macrophage cells through modulation of the TLR4/MyD88 pathways, suggesting that Shinbaro3 is a novel anti-inflammatory therapeutic candidate in the field of pharmacopuncture.

## 1. Introduction

First introduced in Korea in the year 1967, pharmacopuncture is an acupuncture treatment modality that involves the stimulation of acupoints with herbal extracts, rather than with conventional acupuncture needles. The aim is to induce a pharmacological effect of the extracts, in addition to the physical stimulation of conventional acupuncture [1]. Specific subtypes of the technique include *Pal-Kang* (eight principles) pharmacopuncture, monoherbal medicine pharmacopuncture, and mixed herbal medicine pharmacopuncture. These interventions are also currently practised in Europe, within the field of homeopathic medicine [2]. A benefit of pharmacopuncture over the conventional form of acupuncture is the immediacy of the effect, since a small volume of extract is injected directly to stimulate certain acupoints. This method can be useful in patients who experience difficulties in taking herbal medications per os. A diverse range of extracts for pharmacopunctural use is presently under development. Currently, formulations based on *Rehmannia glutinosa*, wild ginseng, *Astragalus propinquus*, and bee venom are in clinical use. Their pharmacopunctural effects against medical conditions such as osteoarthritis, obesity, and cancer are currently under investigation [3–8].

RETRACTED

*Harpagophytum procumbens* is an autogenous species from southern Africa, where the plant has been historically used to treat various conditions, such as fever and rheumatic arthritis [9]. The pharmacological activities of *H. procumbens*, including its anti-inflammatory, analgesic, antioxidative, antiosteoporotic, and antitumour effects, have been described in a number of scientific studies [10–12]. In addition, the signalling pathways involved in the pharmacologic effects of *H. procumbens* and its crude extract have been thoroughly investigated [13, 14].

To enhance its efficacy and absorbance rate of *H. procumbens*, roots of *H. procumbens* var. *sublobatum* (Engl.) Stapf, also known as devil's claw, were alkaline-hydrolysed during the development of the Shinbaro3 formulation. The process of hydrolysis cleaves harpagoside, a known index compound of *H. procumbens*, into two specific molecules, harpagide and cinnamic acid, allowing the induction of their combined effects. A recent study on the standardization of Shinbaro3 reported harpagide and cinnamic acid as two of its index compounds [15]. According to a survey of pharmacopuncture use at an oriental medical hospital for 4 years, Shinbaro3 has been used 3.5% (*n* = 1137/32947) for inpatients and 1.6% (*n* = 4550/289860) for outpatients [16]. Harpagide, one of the active constituents of Shinbaro3, has been shown to exhibit antiosteoporotic properties, both in MC3T3-E1 cells *in vitro* and in an ovariectomized (OVX) mouse model *in vivo* [17].

The human homologue of *Drosophila* toll (hToll), which belongs to the toll-like receptor (TLR) family, plays an important role in the host defence system [18]. Among the different subtypes of TLRs, TLR4 is known to specifically mediate the innate immune response involved in various inflammatory disorders. The activation of the TLR4-mediated signalling pathway upon lipopolysaccharide (LPS) stimulation sends downstream signals through a MyD88- or TRIF-dependent pathway. These signals upregulate the expression of inflammatory cytokines and mediators, resulting in diverse immunological outcomes. Hirotani et al. reported that 80 genes out of 1055 were regulated by either MyD88 or TRIF. Notably, the genes regulated by MyD88 were expressed more rapidly following LPS stimulation than those regulated by TRIF [19].

RETRACTED

Of the 1055 genes that were responsive to LPS stimulation, only 21.5% was found to be dependent on MyD88, while 74.7% was regulated by TRIF. Because TRIF-dependent signalling accounts for more than 70% of all LPS-induced genes, and genes modulated through a TRIF-dependent mechanism contribute significantly to endotoxin lethality, a rational strategy for the development of anti-inflammatory compounds may be to target the TRIF-dependent pathway [20–24].

Thus, any potential anti-inflammatory therapeutic effects mediated by MyD88- and/or TRIF-dependent pathways warrant special investigation. While there have been a number of studies demonstrating the effects of *H. procumbens* on the MyD88-dependent pathway, its potential effects on the TRIF-dependent pathway are still unclear and require further investigation [25]. In this study, the anti-inflammatory effects of Shinbaro3, a pharmacopuncture formulation derived from *H. procumbens*, mediated via MyD88- and TRIF-dependent pathways were investigated in LPS-stimulated RAW 264.7 cells.

## 2. Material and Methods

### 2.1. Preparation of Shinbaro3

Radices of *H. procumbens*, also known as devil's claw, were inspected and approved by the Korean Ministry of Food and Drug Safety (KFDA) (Seoul, Korea). *H. procumbens* (300 g) was boiled in 3 L of 70% ethanol at 85°C for 3 h. The aqueous component of the decoction was then evaporated, and the remaining material was dissolved in 1 L of 80% ethanol. After precipitation at 4°C for 2 h, ethanol was added to obtain a final concentration of 90%.

After vaporization, the resulting powder was dissolved in water (200 mL). The solution was subsequently hydrolysed by the addition of 1 N NaOH for 24 h. Following hydrolysis, the solution was adjusted to pH 7.2 with 1 N NaCl. Finally, the solution was freeze-dried after additional vaporization and stored at −80°C; the powdered product (Shinbaro3) was dissolved in distilled water for use in the assays.

### 2.2. HPLC Fingerprinting of Shinbaro3

Harpagoside (5~500 *μ*g/mL), harpagide (1~100 *μ*g/mL), and cinnamic acid (5 ~ 100 *μ*g/mL) standards were dissolved in 50% methanol. Stock samples of *H. procumbens* extract and Shinbaro3 (hydrolysed *H. procumbens*) were each brought to a concentration of 1 mg/mL for analysis.

High-performance liquid chromatography (LCMS-2020 Shimadzu, ODS C18, 150 × 4.6 mm i.d., 5 *μ*m, Agilent) analysis of harpagoside (*t*_R_ 14.2 min) was performed with 50% methanol: flow rate; 1.5 mL/min, column temperature; 35°C, wavelength; 278 nm, and detector; UV. Harpagide (*t*_R_ 15.0 min) determination was performed using an H_2_O- (0.1% TFA-) acetonitrile (0.1% TFA) gradient (97: 3, 0 → 0 min–90: 10, 0 → 10 min–77: 33, 10 → 20 min–20: 80, 20 → 25 min–20: 80, 25 → 30 min–97: 3, 30 → 31 min–973, 31 → 40 min; total time of 40 min, flow rate: 0.4 mL/min, column temperature: 40°C, detector: MS detector (SIM (+), *m/z* 387). Cinnamic acid fingerprinting (ODS C18, 150 × 4.6 mm i.d., 5 *μ*m, Agilent) was performed with acetonitrile: 1% acetic acid-distilled water (22 : 78) (solvents were used after degassing via ultrasonication), flow rate: 1 mL/min, column temperature: 35°C, wavelength: 280 nm, detector: UV).

RETRACTED

### 2.3. Chemicals and Reagents

LPS (*E. coli* 0111: B4), 3-(4,5-dimethylthiazol-2-yl)-2,5-diphenyltetrazolium bromide (MTT), sulfanilamide, N-(1-naphthyl)-ethylenediamine dihydrochloride, dimethyl sulfoxide (DMSO), harpagoside, cinnamic acid, and TAK-242 were purchased from Sigma-Aldrich (St. Louis, MO, USA). Harpagide was purchased from Chengdu Biopurify Phytochemicals Ltd. (Chengdu, China). Dulbecco's modified Eagle's medium (DMEM), foetal bovine serum (FBS), and an antibiotic-antimycotic solution were purchased from Invitrogen Co. (Grand Island, NY, USA). A sodium nitrite solution was purchased from Fluka (Buchs, Switzerland). Phosphoric acid was purchased from Junsei (Tokyo, Japan). Gene-specific primers were synthesized by Bioneer (Daejeon, Korea). AMV reverse transcriptase, a dNTP mixture, random primers, RNasin, and Taq polymerase were purchased from Promega (Madison, WI, USA). Goat anti-mouse IgG-HRP, goat anti-rabbit IgG-HRP, goat anti-goat IgG-HRP, and antibodies specific for iNOS, COX-2, IL-1*β*, NF-*κ*B p50, NF-*κ*B p65, IKK-*α*/*β*, p-IKK-*α*/*β*, ERK1/2, p-ERK1/2, IRF3, STAT1, p-STAT1, JAK1, and *β*-actin were purchased from Santa Cruz Biotechnology Inc. (Santa Cruz, CA, USA). Antibodies against TNF-*α*, I*κ*B-*α*, p-I*κ*B-*α*, SAPK/JNK, p-SAPK/JNK, p38, p-p38, p-JAK1, p-IRF3, INF-*β*, TLR4, and Myd88 were purchased from Cell Signaling Technology (Beverly, MA, USA).

### 2.4. Cell Lines and Cell Culture

The RAW 264.7 murine macrophage cell line was purchased from American Type Cell Culture (ATCC) (Rockville, MD, USA). The cells were grown in DMEM supplemented with 10% foetal bovine serum (FBS) and 1% antibiotic-antimycotic solution (100 U/mL penicillin G sodium, 100 *μ*g/mL streptomycin sulphate, and 0.25 *μ*g/mL amphotericin B) to a subconfluent density. The cells were cultured at 37°C in a humidified incubator in an atmosphere of 5% CO_2_.

### 2.5. Measurement of Nitric Oxide (NO)

NO generated in the culture medium was measured with the Griess reagent (0.1% N-(1-naphthyl) ethylenediamide dihydrochloride and 1% sulfanilamide in 5% phosphoric acid); NO production was determined directly from this measurement. Briefly, RAW 264.7 cells were seeded in 24-well plates at a density of 2 × 10^5^ cells/mL and then incubated at 37°C in a 5% CO_2_ incubator for 24 h. The cells were subsequently washed with phosphate-buffered saline (PBS), resuspended in fresh medium without FBS, and pretreated with Shinbaro3 or *H. procumbens* extract at different concentrations (200, 400, 800, and 1000 *μ*g/mL) or with vehicle. After incubation for 1 h at 37°C, the cells were stimulated with LPS (1 *μ*g/mL) or vehicle for 20 h. Unstimulated cells were used as a control. A 100 *μ*L aliquot of the supernatant from each well was then transferred to a 96-well plate, and the Griess reagent (180 *μ*L) was added. The absorbance of each well was measured at 540 nm in a microplate reader. The concentration of nitrite in the samples was calculated from a standard curve of sodium nitrite concentrations.

RETRACTED

### 2.6. 3-[4,5-Dimethylthiazol]-2,5-Diphenyltetrazolium Bromide Assay (MTT Assay) for Cell Viability

The colourimetric MTT assay was conducted to examine cell viability. Following 20 h treatment with Shinbaro3 or *H. procumbens* in presence of LPS, MTT solution was added to the culture medium at a final concentration of 500 *μ*g/mL. After 4 h of incubation at 37°C, the medium was discarded, and the formazan blue salt that had formed was dissolved in DMSO (1 mL). A 100 *μ*L aliquot of the supernatant from each well was subsequently transferred to a 96-well plate, and the absorbance was read at 570 nm in an ELISA microplate reader. The percentage of cell survival (%) was calculated relative to the LPS (+) group.

### 2.7. Secreted Embryonic Alkaline Phosphatase (SEAP) Reporter Gene Assay

To investigate the effects of Shinbaro3 on the activation of NF-*κ*B, a reporter gene assay was performed following a previously described method, with some modifications [26]. Cells were pretreated with Shinbaro3 and then stimulated with LPS for an additional 6 h. Next, the culture supernatants were heated at 65°C for 5 min and reacted with SEAP assay buffer [2 M diethanolamine, 1 mM MgCl_2_, and 500 *μ*M 4-methylumbelliferyl phosphate (MUP)] for 1 h in the dark at 37°C. Fluorescence from the SEAP/MUP reaction was measured in relative fluorescence units using a 96-well plate fluorometer, with excitation at 360 nm and emission at 449 nm and was normalized to the protein concentration. Data are presented relative to vehicle-treated control cells without LPS stimulation.

RETRACTED

### 2.8. Western Blot Analysis

RAW 264.7 cells were treated with 150, 300, or 450 *μ*g/mL of Shinbaro3 or vehicle and then stimulated with LPS for various lengths of time (between 2 h and 18 h). To prepare whole-cell lysates, the cells were washed twice with ice-cold PBS and solubilized with extraction lysis buffer (250 mM Tris-HCl pH 6.8, 4% SDS, 10% glycerol, 0.006% bromophenol blue, 50 mM sodium fluoride, 5 mM sodium orthovanadate, and 2% 2-mercaptoethanol). Nucleic/cytoplasmic sample was extracted using a commercially available nuclear extract kit (Active Motif, Carlsbad, CA, USA). The lysates were boiled for 20 min at 100°C and then stored at −20°C until further use. The protein concentration was measured via the bicinchoninic acid assay (BCA).

The quantified protein samples (15–40 *μ*g) were subjected to electrophoresis in 8–10% sodium dodecyl sulphate-polyacrylamide gels and subsequently transferred to a polyvinylidene difluoride (PVDF) membrane (Millipore; MA, USA) for 80 min at 100 V. To block nonspecific binding, the membrane was incubated with 5% bovine serum albumin (BSA) in PBST (0.1% Tween-20 in PBS) for 1 h at room temperature. Subsequently, the membrane was washed three times with PBST, incubated overnight at 4°C with each primary antibody, and washed again three times with PBST. The membrane was then incubated for 90 min at room temperature with the corresponding HRP-conjugated secondary antibody (1 : 1000) and washed again three times with PBST. The signals from the reaction with the enhanced chemiluminescence (ECL) Western blotting detection reagent (Lab Frontier, Suwon, Korea) were visualized using an LAS-4000 Imager (Fujifilm Corp., Tokyo, Japan). All blots were assessed of their quantified density (Supplementary 1).

### 2.9. RNA Extraction and Real-Time Reverse Transcriptase-Polymerase Chain Reaction (Real-Time RT-PCR)

RAW 264.7 cells were incubated for 6 h with LPS or vehicle in the presence or absence of Shinbaro3. The total cellular RNA was isolated from cultured RAW 264.7 cells using TRI reagent (Sigma-Aldrich, St. Louis, MO, USA). Total RNA obtained from each sample (1 *μ*g) was reverse-transcribed (RT) using oligo-(dT)_15_ primers and avian myeloblastosis virus (AMV) reverse transcriptase (Promega, Madison, WI, USA). PCR analyses were performed with the prepared cDNA aliquots to detect gene expression using the GeneAmp PCR system 2400 (Applied Biosystems, Foster, CA, USA). The following primers were employed to analyse the expression of the selected mouse genes: iNOS (sense, 5^'^-GGAGCGAGTTGTGGATTGTC-3′; antisense, 5′-GTGAGGGCTTGGCTGAGTGAG-3′), COX-2 (sense, 5′-GAAGTCTTTGGTCTGGTGCCTG-3′; antisense, 5′-GTCTGCTGGTTTGGAATAGTTGC-3′), TNF-*α* (sense, 5′-CTGTAGCCCACGTCGTAGC-3′; antisense, 5′-TTGAGATCCATGCCGTTG-3′), IL-1*β* (sense, 5′-AGTTGACGGACCCCAAAAG-3′; antisense, 5′-AGCTGGATGCTCTCATCAGG-3′), IFN-*β* (sense, 5′-CACAGCCCTCTCCATCAACTA-3′; antisense, 5′-CATTTCCGAATGTTCGTCCT-3′), TLR4 (sense, 5′-CTCTGGGGAGGCACATCTT-3′; antisense, 5′-CTGCTGTTTGCTCAGGATTC-3′), Myd88 (sense, 5′-GCCAGAGTGGAAAGCAGTGT-3′; antisense, 5′-CGTTGGGGCAGTAGCAGATA-3′), and *β*-actin (sense, 5′-AGACTTCGAGCAGGAGATGG-3′; antisense, 5′-ACCGCTCGTTGCCAATAGT-3′).

RETRACTED

The products of reverse transcription (5 *μ*L) were mixed with iQTM SYBR® Green Supermix (Bio-Rad, Hercules, CA, USA) and the primers in a final volume of 20 *μ*L. Real-time PCR was carried out in a MiniOpticon system (Bio-Rad, Hercules, CA, USA) using standard thermal cycling conditions: 20 s at 95°C, followed by 40 cycles of 20 s at 95°C, 20 s at 56°C, 30 s at 72°C, 1 min at 95°C, and 1 min at 55°C. The threshold cycle (C_T_) was calculated using MJ Opticon Monitor software, as the fractional cycle number at which the amount of the amplified target gene reached a fixed threshold. *β*-Actin was used as the reference housekeeping gene.

### 2.10. Statistical Analysis

Each experiment was performed separately three times, and the results are presented as the mean ± standard deviation (SD). The statistical significance of differences between parameters was evaluated via one-way analysis of variance (ANOVA) coupled with Dunnett's *t*-test.

## 3. Results

### 3.1. HPLC Analysis

Figure 1 shows the HPLC chromatograms obtained for *H. procumbens* and Shinbaro3. The HPLC analysis showed that harpagoside was undetectable in Shinbaro3. The concentrations of harpagide (131.99 *μ*g/g) and cinnamic acid (10.15 *μ*g/g) were higher in Shinbaro3 than in the *H. procumbens* extract (Table 1).

### 3.2. Effects of Shinbaro3 on NO Production and Cell Viability

To investigate the effects of Shinbaro3 on the generation of NO by RAW 264.7 cells stimulated with LPS, a nitrate/nitrite colourimetric assay was performed. The cells were pretreated with 200, 400, 800, or 1000 *μ*g/mL of Shinbaro3, *H. procumbens* extract, or vehicle for 1 h and then stimulated with LPS (1 *μ*g/mL) for 20 h. Shinbaro3 significantly inhibited LPS-induced NO generation, and the inhibitory effect of Shinbaro3 was greater than that of the *H. procumbens* extract, with an IC_50_ of 363.21 *μ*g/mL (Figure 2(a)). The selective iNOS inhibitor 2-amino-5,6-dihydro-6-methyl-4H-1,3-thiazine (AMT) was used as a positive control for the inhibition of NO generation [27]. An MTT assay was performed following the treatment of RAW 264.7 cells with Shinbaro3 to verify whether the suppression of NO generation was due to cytotoxicity. However, no significant cytotoxicity was observed at the tested concentrations of Shinbaro3 (Figures 2(b) and 2(c)); additional experiments confirmed that Shinbaro3 did not show any significant cytotoxicity in RAW 264.7 cells at 6, 12, and 24 h exposure (Supplementary 2). Based on these results, subsequent experiments were conducted to examine the anti-inflammatory effects of Shinbaro3 using concentrations of 150, 300, and 450 *μ*g/mL. The results indicated that Shinbaro3 attenuates LPS-induced NO generation in RAW 264.7 cells.

RETRACTED

### 3.3. Effect of Shinbaro3 on Inflammatory Mediator Expression

When macrophages are activated by stimuli such as LPS, the expression of proinflammatory mediators, such as inducible nitric oxide synthase (iNOS), cyclooxygenase-2 (COX-2), tissue necrosis factor-*α* (TNF-*α*), and interleukin-1*β* (IL-1*β*), is upregulated, triggering the progression of numerous inflammatory diseases [28, 29]. Therefore, the anti-inflammatory effects of Shinbaro3 on the expression of various inflammatory mediators in RAW 264.7 cells after LPS stimulation were explored via real-time RT-PCR and Western blotting. Shinbaro3 downregulated iNOS, COX-2, TNF-*α*, and IL-1*β* mRNA levels in a concentration-dependent manner (Figures 3(a) and 3(b)). Similarly, Western blotting analysis showed that iNOS, TNF-*α*, and IL-1*β* protein expression levels were downregulated by Shinbaro3 in a concentration-dependent manner. LPS-induced COX-2 protein expression was suppressed by Shinbaro3 (Figure 3(c)). These findings indicate that Shinbaro3 modulates inflammatory responses by regulating the expression of inflammatory mediators.

### 3.4. Effects of Shinbaro3 on the NF-*κ*B Signalling Pathway

LPS-induced activation of NF-*κ*B, a transcription factor, triggers its translocation into the nucleus, where it binds to specific promoter regions and regulates the expression of a wide variety of inflammatory mediators. To investigate the potential of Shinbaro3 to modulate the NF-*κ*B signalling pathway in RAW 264.7 cells after LPS stimulation, Western blot analysis was performed using antibodies specific for NF-*κ*B p65, NF-*κ*B p50, I*κ*B-*α*, and IKK-*α*/*β*. RAW 264.7 cells were treated with Shinbaro3 and LPS for 2 h. LPS stimulation was found to induce nuclear translocation of p50 and p65 subunits, and Shinbaro3 inhibited LPS-induced translocation of NF-*κ*B subunits in a dose-dependent manner (Figure 4(a)). As expected, the phosphorylation of IKK-*α*/*β* and subsequent degradation of I*κ*B-*α* were observed in RAW cells stimulated with LPS in the cytoplasm. These signalling events were also reversed by Shinbaro3 in a concentration-dependent manner (Figures 4(b) and 4(c)). As an additional readout to determine the modulatory effects of Shinbaro3 on NF-*κ*B transcriptional activity, we conducted a secreted embryonic alkaline phosphatase (SEAP) reporter gene assay. NF-*κ*B activity was increased after LPS stimulation, and Shinbaro3 significantly inhibited this transcriptional activity in a concentration-dependent manner (Figure 4(d)). Overall, these results indicate that regulation of the NF-*κ*B pathway may contribute to the anti-inflammatory effects of Shinbaro3.

RETRACTED

### 3.5. Effects of Shinbaro3 on MAPK Family Pathways

Mitogen-activated protein kinases (MAPKs)—comprising stress-activated protein kinase/c-Jun N-terminal kinase (SAPK/JNK), extracellular signal-regulated protein kinases (ERK1/2), and p38 MAPK—play significant roles in the regulation of the expression of inflammatory mediators, including iNOS in macrophages [30]. To examine the effects of Shinbaro3 on MAPK pathways, Western blotting assays were performed. Cells were treated with LPS (1 *μ*g/mL) and various concentrations of Shinbaro3 for 2 h. While LPS stimulation induced the activation of ERK1/2, SAPK/JNK, and p38 MAPK in RAW 264.7 cells, Shinbaro3 treatment suppressed the LPS-induced phosphorylation of these MAPKs in a concentration-dependent manner (Figure 5). Thus, suppression of MAPK signalling pathways is thought to be partly responsible for the anti-inflammatory effects of Shinbaro3.

### 3.6. Effects of Shinbaro3 on IRF3 and the STAT1 Signalling Pathway

LPS upregulates the expression of IFN-*β*; inhibition of IRF3, downstream of the TLR4-TRIF-dependent signalling pathway, has been shown to downregulate LPS-induced IFN-*β* expression, resulting in amelioration of inflammatory responses [20, 22, 31]. The effect of Shinbaro3 on the LPS-induced activation of IRF3 was explored through immunoblotting. RAW 264.7 cells were treated with various concentrations of Shinbaro3 and LPS (1 *μ*g/mL) for 4 h. As expected, stimulation of RAW 264.7 cells with LPS activated IRF3. In contrast, pretreatment with Shinbaro3 suppressed the LPS-induced activation of IRF3 (Figure 6(a)). In addition, phosphorylation of IRF3 has been known to activate JAK1/STAT1 pathways. As Shinbaro3 was found to suppress IRF3 activation, the effects of Shinbaro3 on JAK1/STAT1 pathways were also examined. The results showed that Shinbaro3 inhibited LPS-induced JAK1/STAT1 activation in a concentration-dependent manner (Figures 6(a)). To investigate the consequences of IRF3 inhibition by Shinbaro3 for IFN-*β* mRNA expression, real-time RT-PCR was performed. While LPS upregulated IFN-*β* mRNA expression, Shinbaro3 inhibited IFN-*β* mRNA expression in a concentration-dependent manner (Figure 6(c)). Consequently, the inhibitory effect of Shinbaro3 on INF-*β* protein expression was also examined. As observed through Western blot, Shinbaro3 suppressed LPS-induced protein expression of INF-*β* in a concentration-dependent manner (Figure 6(b)). To further examine whether Shinbaro3 targets JAK1/STAT1 pathway, additional experiments were conducted where RAW 264.7 cells were stimulated with INF-*β*. As expected, JAK1 and STAT1 were phosphorylated upon INF-*β* stimulation; Shinbaro3 suppressed INF-*β*-induced phosphorylation of JAK1/STAT1 in a concentration-dependent manner (Figure 6(d)). The data demonstrate that Shinbaro3 exerts a suppressive effect on LPS-induced IFN-*β* expression that may be partly due to suppression of the IRF3/STAT1 signalling pathway, and that Shinbaro3 downregulates JAK1/STAT1 pathway, thereby exhibiting anti-inflammatory effects.

RETRACTED

### 3.7. Effects of Shinbaro3 on the TLR4/Myd88 Signalling Pathway

The TLR4 signalling pathway plays a significant role in immune responses. Activation of TLR4 in RAW 264.7 cells following LPS stimulation regulates the NF-*κ*B and MAPK signalling pathways [32, 33]. To further explore the mechanisms responsible for the effects of Shinbaro3 on the TLR4-mediated signalling pathway, TLR4 and Myd88 protein and mRNA expression were analysed via Western blotting and real-time RT-PCR. TLR4 and Myd88 protein and mRNA levels were significantly increased by LPS stimulation. In contrast, Shinbaro3 decreased the expression of TLR4 and Myd88 in a concentration-dependent manner. To evaluate the specificity of the LPS-induced expression of TLR4 and Myd88, we employed a specific TLR4 inhibitor (TAK-242). TAK-242 inhibited TLR4 and Myd88 mRNA expression following LPS stimulation (Figure 7). Taken together, these results suggest that the anti-inflammatory activity of Shinbaro3 depends on the suppression of the TLR4/Myd88 signalling pathway.

## 4. Discussion

Shinbaro3 is derived from *H. procumbens* through the hydrolysis of harpagoside into harpagide and cinnamic acid and is currently used to treat various inflammatory disorders and degenerative musculoskeletal diseases. Although the anti-inflammatory effects of *H. procumbens*, harpagoside, harpagide, and cinnamic acid have been observed in a number of studies, the mechanisms through which these compounds exert their pharmacological effects have so far remained elusive [34–37]. Therefore, the current study explored the effects of Shinbaro3 on the TLR4 signalling pathway, which is one of the most important pathways targeted in anti-inflammatory therapy, and has not been previously investigated in connection with Shinbaro3.

HPLC analysis was performed to determine the concentrations of harpagoside, harpagide, and cinnamic acid in Shinbaro3 and in the *H. procumbens* extract. Harpagoside was not detected in the HPLC chromatogram of Shinbaro3, resulting in a relative increase in the concentrations of harpagide and cinnamic acid (Figure 1).

RETRACTED

NO species play an essential role in the modulation of inflammatory processes. Under physiological conditions, NO sends signals that mediate various cellular functions, suppresses proliferation, and induces apoptosis. Context-sensitive regulation of these processes is crucial to maintain homeostasis. However, excessive generation of NO following uncontrolled iNOS activation may cause gene mutations and cytotoxicity. These pathological changes in body components such as the joints, intestinal epithelium, and pulmonary epithelium may play a role in the tissue damage associated with various diseases, such as arthritis and asthma [38]. Therefore, modulation of NO generation may be a rational strategy for improving anti-inflammatory therapies.

To investigate the effects of Shinbaro3 on NO generation in LPS-stimulated RAW 264.7 cells, nitrite species were examined. Our results suggested that the inhibitory effects of Shinbaro3 on NO production were greater than those of *H. procumbens.* Shinbaro3 inhibited NO generation in a concentration-dependent manner without significant cytotoxicity (IC_50_ = 363.21 *μ*g/mL) (Figure 2(a)). Furthermore, Shinbaro3 was found to suppress the LPS-induced expression of iNOS mRNA and protein in a concentration-dependent manner (Figures 3(a) and 3(c)). These findings are in agreement with a previous report showing that the aqueous extract of *H. procumbens* inhibits iNOS expression in LPS-stimulated L929 murine cells in a dose-dependent manner [39]. Similarly, Kaszkin et al. observed significant suppression of nitrite production and iNOS expression by *H. procumbens* in IL-1*β*-stimulated mesangial cells, using concentrations of 0.3–1.0 mg/mL [40]. Considering these results, the inhibitory effects of Shinbaro3 on NO generation may be attributed to the downregulation of iNOS at both the transcriptional and translational levels.

Cyclooxygenase (COX), a prostaglandin G/H synthase, is expressed as at least two different isozymes. COX-1 is a housekeeping enzyme and is the isoform that is constitutively expressed in most tissues. In contrast, COX-2 is present at considerable levels only at inflammatory sites and is rapidly induced by proinflammatory mediators such as TNF-*α*, IL-1*β*, and IFN-*β*; the expression of COX-2 under physiological conditions is insignificant [28]. In this study, the LPS-induced mRNA expression of COX-2 was found to be suppressed by Shinbaro3 in a concentration-dependent manner (Figure 3(a)); however, no concentration-dependent effect of Shinbaro3 on the protein expression of COX-2 was observed (Figure 3(c)). Consequently, it can be deduced that the inhibition of COX-2 expression by *H. procumbens* may be attributed to the interaction of numerous components.

RETRACTED

In addition to iNOS and COX-2, proinflammatory cytokines such as TNF-*α* and IL-1*β* also play significant roles in the modulation of inflammatory responses. The anti-inflammatory effects of Shinbaro3 on TNF-*α* and IL-1*β* expression by LPS-stimulated RAW 264.7 cells were investigated at both the mRNA and protein levels. As shown in Figures 3(b) and 3(c), Shinbaro3 suppressed TNF-*α* and IL-1*β* mRNA and protein expression in a concentration-dependent manner. In a recent publication, the authors investigated the effects of a crude extract obtained from *H. procumbens* on the expression of 12 individual human inflammatory cytokines by THP-1 human monocytes following KPS stimulation. The results showed that the expression of TNF-*α*, IL-6, IL-8, and IL-1 was downregulated by *H. procumbens* [41]. Similarly, Inaba et al. reported dose-dependent inhibitory effects of *H. procumbens* extract on the expression of inflammatory cytokines (e.g., TNF-*α*, IL-1*β*, and IL-6) in LPS-stimulated mouse macrophages [42]. The results of these studies indicate that Shinbaro3 can act as a potent inhibitor of various inflammatory mediators.

When proinflammatory stimuli activate the IKK complex, I*κ*B-*α* is phosphorylated, selectively ubiquitinated, and then quickly degraded, which in turn controls the activation and nuclear translocation of NF-*κ*B. To investigate whether the NF-*κ*B pathway was involved in the suppressive effects of Shinbaro3 on IL-1*β* and TNF-*α* expression, Western blotting assays were performed. We found that Shinbaro3 suppressed the upregulation of NF-*κ*B subunit expression and inhibited IKK-*α*/*β* activity, thereby preserving I*κ*B-*α* and downregulating the NF-*κ*B pathway. Shinbaro3 also inhibited the LPS-induced increase in NF-*κ*B transcriptional activity in a concentration-dependent manner (Figure 4). The current results are in agreement with a previous report showing that both *H. procumbens* extract and harpagoside suppress the NF-*κ*B pathway as well as iNOS and COX-2 expression [43]. Based on these findings, the anti-inflammatory effects of Shinbaro3 are assumed to include modulation of the NF-*κ*B pathway.

In addition to the NF-*κ*B pathway, the MAPK pathway regulates various inflammatory mediators, such as iNOS and COX-2. Both the NF-*κ*B and MAPK pathways are modulated by TLR4. The findings of the present study demonstrate that Shinbaro3 suppresses the activation of ERK, SAPK/JNK, and p38 in LPS-stimulated RAW 264.7 cells in a dose-dependent manner (Figure 5). These effects may account for the observed suppressive effect of Shinbaro3 on iNOS expression and NO generation. In agreement with these results, Kundu et al. reported that the methanol extract of *H. procumbens* inhibited COX-2 expression *in vivo* by blocking ERK activity in mouse skin stimulated with 12-O-tetradecanoylphorbol-13-acetate (TPA) [44]. Our results imply that the anti-inflammatory effects of Shinbaro3 may be associated with downregulation of MAPK signalling through a Myd88-dependent pathway.

RETRACTED

After stimulation with a TLR4 agonist, activated IRF3 is translocated into the nucleus and promotes the expression of type 1 interferons (IFNs); expression of IFN-mediated genes, such as iNOS, IL-6, and monocyte chemoattractant protein-1 (MCP-1), occurs subsequently [45–47]. The generation of NO has been reported to be directly dependent on the IRF3/IFN-*β* pathway [20]. Toshchakov et al. reported that *E. coli* LPS dramatically induced IFN-*β* expression in a TLR4-dependent manner, leading to phosphorylation of STAT1 [48]. According to the current results, Shinbaro3 inhibits IRF3 activation in LPS-stimulated RAW 264.7 cells, an effect that is related to the downregulated expression of IFN-*β* protein and mRNA and subsequent suppression of the JAK1/STAT1 pathway. Phosphorylation of JAK1/STAT1 was suppressed by Shinbaro3 after IFN-*β* stimulation (Figure 6). These findings demonstrate that Shinbaro3 modulates inflammatory responses by regulating a TRIF-dependent pathway. In addition, Shinbaro3 suppresses the upregulation of TLR4 and Myd88 expression in response to LPS stimulation in a concentration-dependent manner (Figure 7). The current findings demonstrate that Shinbaro3 exerts its anti-inflammatory effect via regulating the TLR4-related signalling pathway.

Major constituents of *H. procumbens* include harpagoside, harpagide, 8-O-p-coumaroyl harpagide, 8-feruloylharpagide, procumbide, and phesnylethanoid glycoside verbascoside; the pharmacological activity of the plant is mainly attributed to harpagoside [9]. Based on previous researches, harpagoside is known to target BMP2/Wnt signaling [12] and NF-kappaB pathway [43]; it also modulates various mediators such as TNF-alpha [14], COX-2 [37], and iNOS [43]. Natural compounds with anti-inflammatory activity are often reported of their multitargeting nature [49], and so is believed to be true with *H. procumbens*. While Shinbaro3, a hydrolysed variant of *H. procumbens*, similarly shares such characteristics, its suppressive activity on NO generation has been found to be superior having an equivalent amount of harpagoside, harpagide, or cinnamic acid (Supplementary 3), whether such phenomenon comes from synergism of various constituents or the hydrolysis process is needed to be investigated in future studies.

RETRACTED

Pharmacopuncture is a type of acupuncture technique where the herbal extract is injected into acupoints [1]. Shinbaro3 was developed as one of the pharmacopuncture agents, and it has been widely used for musculoskeletal disorders, as reported by a survey among Korean medical doctors [16]. While Shinbaro3 has been shown to exert clinical effects in such patients, its use has been mainly based on empirical results. A regular dose of Shinbaro3 for human use was reported to be around 0.12 mg/60 kg [16]. Previously conducted scientific studies on Shinbaro3 mostly reported of toxicity data in rats and beagles [50, 51]. Even though Shinbaro3 was developed from hydrolysed *H. procumbens*, its pharmacologic activity may differ from *H. procumbens*, as demonstrated earlier. More rigorous studies on pharmacologic actions of Shinbaro3 are warranted in future. Moreover, synergistic effect brought by a pharmacologic agent and physical stimulation of the acupuncture needle will be an interesting topic in the field.

The aim of the present study was to investigate the mechanism by which Shinbaro3 exerts anti-inflammatory effects. Based on the current results, Shinbaro3 is believed to modulate (1) MAPKs, (2) NF-*κ*B pathways (both involved with MyD88-dependent signalling), and (3) IRF3/JAK1/STAT1 pathway—involved with TRIF-dependent signalling. Based on these combined effects, Shinbaro3 may be valuable as a novel candidate in the search for potent anti-inflammatory therapeutic compounds.

## Figures and Tables

**Figure 1:** HPLC chromatograms of *H. procumbens* extract and Shinbaro3. HPLC chromatogram peaks corresponding to (a) harpagoside, (b) harpagide, and (c) cinnamic acid in *H. procumbens* extract (before hydrolysis) and alkaline-hydrolysed Shinbaro3 (after hydrolysis).

**Figure 2:** Effects of Shinbaro3 on NO production in LPS-stimulated RAW 264.7 macrophage cells. (a) RAW 264.7 cells were stimulated with LPS (1 *μ*g/mL) for 20 h in the absence or presence of Shinbaro3 (after hydrolysis) or *H. procumbens* extract (before hydrolysis) (200, 400, 800, or 1000 *μ*g/mL). The nitrite concentration in the supernatant was detected via the Griess reaction. (b) Cell viability upon Shinbaro3 or *H. procumbens* treatment for 20 h was evaluated using the MTT assay, as described in Materials and Methods. (c) Morphological changes produced by Shinbaro3 in LPS-stimulated macrophages, photographed with an inverted phase-contrast microscope. Data are presented as the mean ± SD (*n* = 3). ^∗^*p* < 0.05, ^∗∗^*p* < 0.01, and ^∗∗∗^*p* < 0.001 versus LPS treatment alone.

RETRACTED

**Figure 3:** Effects of Shinbaro3 on the expression of inflammatory mediators in LPS-stimulated RAW 264.7 macrophage cells. RAW 264.7 cells were treated with LPS (1 *μ*g/mL) and Shinbaro3 (150, 300, and 450 *μ*g/mL) for 6 h to investigate mRNA expression (a, b) or 18 h to investigate protein expression (c). iNOS, COX-2, TNF-*α* and IL-1*β* mRNA, and protein expression levels were then analysed in real-time RT-PCR and Western blot assays, respectively. The results were normalized using *β*-actin as an internal control. Data are presented as the mean ± SD (*n* = 3). ^∗^*p* < 0.05, ^∗∗^*p* < 0.01, and ^∗∗∗^*p* < 0.001 versus LPS treatment alone.

**Figure 4:** Effects of Shinbaro3 on NF-*κ*B activation in LPS-stimulated RAW 264.7 cells. RAW 264.7 cells were treated with LPS (1 *μ*g/mL) and Shinbaro3 (150, 300, and 450 *μ*g/mL) for 2 h to investigate protein expression or 6 h for SEAP analysis. Nuclear and cytoplasm extracts were analysed via Western blotting. (a–c) The expression levels of NF-*κ*B (p65 and p50 subunits) (nuclear fraction), p-I*κ*B-*α*, IκB-*α*, p-IKK-*α*, and IKK-*α* (cytoplasmic fraction) were measured using specific antibodies. Lamin B1 (nuclear fraction) and *β*-actin (cytoplasmic fraction) were used as an internal control. The data are representative of three separate experiments. (d) Effects of Shinbaro3 on NF-*κ*B transcriptional activity were assessed though a reporter gene assay. Relative fluorescence units (RFU) were measured by using a fluorometer for secreted alkaline phosphatase activity (SEAP). The data are expressed as the mean ± SD (*n* = 3). ^∗^*p* < 0.05, ^∗∗^*p* < 0.01, and ^∗∗∗^*p* < 0.001 versus LPS treatment alone.

**Figure 5:** Effects of Shinbaro3 on MAPK phosphorylation in LPS-stimulated RAW 264.7 cells. RAW 264.7 cells were treated with LPS (1 *μ*g/mL) and Shinbaro3 (150, 300, and 450 *μ*g/mL) for 2 h. Total cell lysates were analysed via Western blotting using antiphospho-ERK1/2, antiphospho-SAPK/JNK, and antiphospho-p38 antibodies. *β*-Actin was used as an internal control. The data are representative of three separate experiments.

**Figure 6:** Effects of Shinbaro3 on the IRF3/STAT1 signalling pathway in LPS-stimulated RAW 264.7 cells. RAW 264.7 cells were treated with LPS (1 *μ*g/mL) and Shinbaro3 (150, 300, and 450 *μ*g/mL) for 4 h. The expression levels of (a) IRF3, STAT1, JAK1, and their phosphorylated forms were detected with specific antibodies. *β*-Actin was used as an internal control. The data are representative of three separate experiments. (b) Protein expression of INF-*β* was assessed in RAW 264.7 cells under the above condition. (c) RAW 264.7 cells were treated with LPS (1 *μ*g/mL) and Shinbaro3 (150, 300, and 450 *μ*g/mL) for 6 h. Expression of IFN-*β* was investigated with real-time RT-PCR as described in Materials and Methods. (d) RAW 264.7 cells were stimulated with Shinbaro3 (150, 300, and 450 *μ*g/mL) in presence of IFN-*β* (100 U/mL) for 4 h. Protein expression of JAK1 and STAT1 and their phosphorylated forms were detected. The data are expressed as the mean ± SD (*n* = 3). ^∗^*p* < 0.05, ^∗∗^*p* < 0.01, and ^∗∗∗^*p* < 0.001 versus LPS treatment alone.

RETRACTED

**Figure 7:** Effects of Shinbaro3 on the TLR4/Myd88 signalling pathway in LPS-stimulated RAW 264.7 cells. RAW 264.7 cells were treated with LPS (1 *μ*g/mL) and Shinbaro3 (150, 300, and 450 *μ*g/mL) for 6 h. (a, b) TLR4 and (c, d) Myd88 protein and mRNA expression levels were analysed via Western blotting and real-time RT-PCR, respectively. The results were normalized using *β*-actin as an internal control. The data are presented as the mean ± SD (*n* = 3). ^∗^*p* < 0.05, ^∗∗^*p* < 0.01, and ^∗∗∗^*p* < 0.001 versus LPS treatment alone.

**Figure 8:** Overview of the TLR4 signalling pathway. The mechanisms underlying the inhibitory effects of Shinbaro3 on the LPS-induced inflammatory response.

**Table 1:** Quantities of compounds present in *H. procumbens* extract and Shinbaro3.

Compound	Retention time (min)	Regression equation	*r* ^2^	Concentration (*μ*g/g)	
				*H. procumbens*	Shinbaro3
Harpagoside	14.2	*y* = 3729.9*x* − 4852.3	1.0000	77.41	0.00
Harpagide	15.0	*y* = 67561*x* + 750223	0.9847	58.04	131.99
Cinnamic acid	32.1	*y* = 10926*x* − 3084.1	0.9999	0.0032	10.15

## Supplementary Materials

Supplementary Materials Supplemental Figure 1: all Western blots were assessed of their quantified density. Figure 3 (c): effects of Shinbaro3 on the expression of inflammatory mediators in LPS-stimulated RAW 264.7 macrophage cells. (Figure 3c) RAW 264.7 cells were treated with LPS (1 *μ*g/mL) and Shinbaro3 (150, 300, and 450 μg/mL) for 18 h to investigate protein expression. iNOS, COX-2, TNF-*α*, and IL-1*β* mRNA and protein expression levels were then analysed in Western blot assays. *β*-Actin was used as an internal control. The data are representative of three separate experiments. Figure 4: effects of Shinbaro3 on NF-*κ*B activation in LPS-stimulated RAW 264.7 cells. RAW 264.7 cells were treated with LPS (1 *μ*g/mL) and Shinbaro3 (150, 300, and 450 *μ*g/mL) for 2 h to investigate protein expression. Nuclear and cytoplasm extracts were analysed via Western blotting. (Figures 4a–4c) The expression level of NF-*κ*B (p65 and p50 subunits) (nuclear fraction), p-I*κ*B-*α*, I*κ*B-*α*, and p-IKK-*α* (cytoplasmic fraction) were measured using specific antibodies. Lamin B1 (nuclear fraction) and *β*-actin (cytoplasmic fraction) were used as an internal control. The data are representative of three separate experiments. Figure 5: effects of Shinbaro3 on MAPK phosphorylation in LPS-stimulated RAW 264.7 cells. RAW 264.7 cells were treated with LPS (1 *μ*g/mL) and Shinbaro3 (150, 300, and 450 *μ*g/mL) for 2 h. Total cell lysates were analysed via Western blotting using antiphospho-ERK1/2, antiphospho-SAPK/JNK, and antiphospho-p38 antibodies. *β*-Actin was used as an internal control. The data are representative of three separate experiments. Figure 6: effects of Shinbaro3 on the IRF3/STAT1 signalling pathway in LPS-stimulated RAW 264.7 cells. RAW 264.7 cells were treated with LPS (1 *μ*g/mL) and Shinbaro3 (150, 300, and 450 *μ*g/mL) for 4 h. The expression levels of (a) IRF3, STAT1, JAK1 and their phosphorylated forms were detected with specific antibodies. (b) Protein expression of INF-*β* was assessed in RAW 264.7 cells under the above condition. (d) RAW 264.7 cells were stimulated with Shinbaro3 (150, 300, and 450 *μ*g/mL) in the presence of IFN-*β* (100 U/mL) for 4 h. Protein expression of JAK1 and STAT1 and their phosphorylated forms were detected. *β*-Actin was used as an internal control. The data are representative of three separate experiments. Figure 7: effects of Shinbaro3 on the TLR4/Myd88 signalling pathway in LPS-stimulated RAW 264.7 cells. RAW 264.7 cells were treated with LPS (1 *μ*g/mL) and Shinbaro3 (150, 300, and 450 *μ*g/mL) for 6 h. (a) TLR4 and (c) Myd88 protein expression levels were analysed via Western blotting. *β*-Actin was used as an internal control. The data are representative of three separate experiments. Supplemental Figure 2: Shinbaro3 did not show any significant cytotoxicity in RAW 264.7 cells at 6, 12, and 24 h exposure. Cell viability upon Shinbaro3 or *H. procumbens* treatment for 6, 12, and 24 h was evaluated using the MTT assay, as described in Materials and Methods. Data are presented as the mean ± SD (*n* = 3). Supplemental Figure 3: NO generation and cell viability have been found to be superior to an equivalent amount of harpagoside, harpagide, or cinnamic acid in LPS-stimulated RAW 264.7 macrophage cells. (a) Raw 264.7 cells were stimulated with LPS (1 *μ*g/mL) for 20 h in the absence or presence of harpagoside, harpagide, or cinnamic acid (200, 400, 800, or 1000 *μ*g/mL). The nitrite concentration in the supernatant was detected via the Griess reaction. (b) Cell viability upon harpagoside, harpagide, or cinnamic acid treatment for 20 h was evaluated using the MTT assay, as described in Materials and Methods. Data are presented as the mean ± SD (*n* = 3).

RETRACTED

## References

[1] Park J., Lee H., Shin B.-C., Lee M. S., Kim B., Kim J.-I. (2016). Pharmacopuncture in Korea: a systematic review and meta-analysis of randomized controlled trials. *Evidence-Based Complementary and Alternative Medicine*.

[2] Frass M., Friehs H., Thallinger C. (2015). Influence of adjunctive classical homeopathy on global health status and subjective wellbeing in cancer patients – a pragmatic randomized controlled trial. *Complementary Therapies in Medicine*.

[3] Cheon S., Zhang X., Lee I.-S., Cho S.-H., Chae Y., Lee H. (2014). Pharmacopuncture for cancer care: a systematic review. *Evidence-Based Complementary and Alternative Medicine*.

[4] Kang K.-H., Lee K.-H., Yoon H.-M., Jang K.-J. (2012). Rehmannia glutinosa pharmacopuncture solution regulates functional activation, Fc*ε*RI expression, and signaling events in mast cells. *Journal of Pharmacopuncture*.

[5] Lee S.-H., Kwon G.-S., Kang M.-S., Yoon H.-M., Kim C.-H. (2012). Comparative study on the effects of bee venom pharmacopuncture according to the treatment method for knee osteoarthritis. *Journal of Pharmacopuncture*.

[6] Park J.-W., Jeon J.-H., Yoon J. (2012). Effects of sweet bee venom pharmacopuncture treatment for chemotherapy-induced peripheral neuropathy. a case series. *Integrative Cancer Therapies*.

[7] Nam M.-H., Lee S.-W., Na H.-Y. (2016). Herbal acupuncture for the treatment of obesity. *Journal of Acupuncture and Meridian Studies*.

[8] Yook T., Yu J., Lee H. (2009). Comparing the effects of distilled *Rehmannia glutinosa*, *wild ginseng* and *Astragali Radix* pharmacopuncture with heart rate variability (HRV): a randomized, sham-controlled and double-blind clinical trial. *Journal of Acupuncture and Meridian Studies*.

[9] Georgiev M. I., Ivanovska N., Alipieva K., Dimitrova P., Verpoorte R. (2013). Harpagoside: from Kalahari Desert to pharmacy shelf. *Phytochemistry*.

[10] McGregor G., Fiebich B., Wartenberg A., Brien S., Lewith G., Wegener T. (2005). Devil’s claw (*Harpagophytum procumbens*): an anti-inflammatory herb with therapeutic potential. *Phytochemistry Reviews*.

[11] Mncwangi N., Chen W., Vermaak I., Viljoen A. M., Gericke N. (2012). Devil’s claw—a review of the ethnobotany, phytochemistry and biological activity of *Harpagophytum procumbens*. *Journal of Ethnopharmacology*.

[12] Chung H.-J., Kim W. K., Oh J. (2017). Anti-osteoporotic activity of harpagoside by upregulation of the BMP2 and Wnt signaling pathways in osteoblasts and suppression of differentiation in osteoclasts. *Journal of Natural Products*.

RETRACTED

[13] Kim T. K., Park K. S. (2015). Inhibitory effects of harpagoside on TNF-*α*-induced pro-inflammatory adipokine expression through PPAR-*γ* activation in 3T3-L1 adipocytes. *Cytokine*.

[14] Schopohl P., Gruneberg P., Melzig M. F. (2016). The influence of harpagoside and harpagide on TNF*α*-secretion and cell adhesion molecule mRNA-expression in IFN*γ*/LPS-stimulated THP-1 cells. *Fitoterapia*.

[15] Lee J.-H., Lee J.-W., Kim M.-J., Kim E.-J., Lee I.-H. (2015). Identification of novel standard compounds for standardization of Sinbaro3 pharmacopuncture. *Journal of Korean Medicine Rehabilitation*.

[16] Lee Y. J., Shin J.-S., Lee J. (2016). Usage report of pharmacopuncture in musculoskeletal patients visiting Korean medicine hospitals and clinics in Korea. *BMC Complementary and Alternative Medicine*.

[17] Chung H.-J., Kim W. K., Park H. J. (2016). Anti-osteoporotic activity of harpagide by regulation of bone formation in osteoblast cell culture and ovariectomy-induced bone loss mouse models. *Journal of Ethnopharmacology*.

[18] Takeda K., Akira S. (2004). TLR Signaling Pathways. *Seminars in Immunology*.

[19] Hirotani T., Yamamoto M., Kumagai Y. (2005). Regulation of lipopolysaccharide-inducible genes by MyD88 and toll/IL-1 domain containing adaptor inducing IFN-*β*. *Biochemical and Biophysical Research Communications*.

[20] Abe M., Matsuda M., Kobayashi H. (2008). Effects of statins on adipose tissue inflammation: their inhibitory effect on MyD88-independent IRF3/IFN-*β* pathway in macrophages. *Arteriosclerosis, Thrombosis, and Vascular Biology*.

[21] Björkbacka H., Fitzgerald K. A., Huet F. (2004). The induction of macrophage gene expression by LPS predominantly utilizes Myd88-independent signaling cascades. *Physiological Genomics*.

[22] Kim M. H., Yoo D. S., Lee S. Y. (2011). The TRIF/TBK1/IRF-3 activation pathway is the primary inhibitory target of resveratrol, contributing to its broad-spectrum anti-inflammatory effects. *Pharmazie*.

[23] Lee J. K., Kim S. Y., Kim Y. S., Lee W.-H., Hwang D. H., Lee J. Y. (2009). Suppression of the TRIF-dependent signaling pathway of toll-like receptors by luteolin. *Biochemical Pharmacology*.

[24] Shaik-Dasthagirisaheb Y. B., Huang N., Gibson F. C. (2014). Inflammatory response to *Porphyromonas gingivalis* partially requires interferon regulatory factor (IRF) 3. *Innate Immunity*.

[25] Jiang J., Kang T. B., Oh N. H., Kim T. J., Lee K. H. (2013). Indole-3-carbinol inhibits LPS-induced inflammatory response by blocking TRIF-dependent signaling pathway in macrophages. *Food and Chemical Toxicology*.

[26] Moon K.-Y., Hahn B.-S., Lee J., Kim Y. S. (2001). A cell-based assay system for monitoring NF-*κ*B activity in human HaCat transfectant cells. *Analytical Biochemistry*.

RETRACTED

[27] Nakane M., Klinghofer V., Kuk J. E. (1995). Novel potent and selective inhibitors of inducible nitric oxide synthase. *Molecular Pharmacology*.

[28] Gilroy D. W., Colville-Nash P. R. (2000). New insights into the role of COX 2 in inflammation. *Journal of Molecular Medicine*.

[29] Kim J.-B., Han A.-R., Park E.-Y. (2007). Inhibition of LPS-induced iNOS, COX-2 and cytokines expression by poncirin through the NF-*κ*B inactivation in RAW 264.7 macrophage cells. *Biological and Pharmaceutical Bulletin*.

[30] Zhou H. Y., Shin E. M., Guo L. Y. (2008). Anti-inflammatory activity of 4-methoxyhonokiol is a function of the inhibition of iNOS and COX-2 expression in RAW 264.7 macrophages via NF-*κ*B, JNK and p38 MAPK inactivation. *European Journal of Pharmacology*.

[31] Sugiyama Y., Kakoi K., Kimura A. (2012). Smad2 and Smad3 are redundantly essential for the suppression of iNOS synthesis in macrophages by regulating IRF3 and STAT1 pathways. *International Immunology*.

[32] Gorina R., Font-Nieves M., Márquez-Kisinousky L., Santalucia T., Planas A. M. (2011). Astrocyte TLR4 activation induces a proinflammatory environment through the interplay between MyD88-dependent NF*κ*B signaling, MAPK, and Jak1/Stat1 pathways. *Glia*.

[33] Liu T., Gao Y. J., Ji P. R. (2012). Emerging role of toll-like receptors in the control of pain and itch. *Neuroscience Bulletin*.

[34] Anauate M. C., Torres L. M., de Mello S. B. V. (2010). Effect of isolated fractions of *Harpagophytum procumbens* D.C. (devil's claw) on COX-1, COX-2 activity and nitric oxide production on whole-blood assay. *Phytotherapy Research*.

[35] Hadjipavlou-Litina D., Pontiki E., Armstrong D. (2015). Aryl-acetic and cinnamic acids as lipoxygenase inhibitors with antioxidant, anti-inflammatory, and anticancer activity. *Advanced Protocols in Oxidative Stress III. Methods in Molecular Biology (Methods and Protocols)*.

[36] Liu L., Hudgins W. R., Shack S., Yin M. Q., Samid D. (1995). Cinnamic acid: a natural product with potential use in cancer intervention. *International Journal of Cancer*.

[37] Zhang L., Feng L., Jia Q. (2011). Effects of *β*-glucosidase hydrolyzed products of harpagide and harpagoside on cyclooxygenase-2 (COX-2) in vitro. *Bioorganic & Medicinal Chemistry*.

[38] Sharma J., Al-Omran A., Parvathy S. (2007). Role of nitric oxide in inflammatory diseases. *Inflammopharmacology*.

[39] Jang M. H., Lim S., Han S. M. (2003). *Harpagophytum procumbens* suppresses lipopolysaccharide-stimulated expressions of cyclooxygenase-2 and inducible nitric oxide synthase in fibroblast cell line L929. *Journal of Pharmacological Sciences*.

RETRACTED

[40] Kaszkin M., Beck K., Koch E., Erdelmeier S. K., Pfeilschifter J., Loew D. (2004). Downregulation of iNOS expression in rat mesangial cells by special extracts of *Harpagophytum procumbens* derives from harpagoside-dependent and independent effects. *Phytomedicine*.

[41] Hostanska K., Melzer J., Rostock M., Suter A., Saller R. (2014). Alteration of anti-inflammatory activity of Harpagophytum procumbens (devil’s claw) extract after external metabolic activation with S9 mix. *Journal of Pharmacy and Pharmacology*.

[42] Inaba K., Murata K., Naruto S., Matsuda H. (2010). Inhibitory effects of devil’s claw (secondary root of *Harpagophytum procumbens*) extract and harpagoside on cytokine production in mouse macrophages. *Journal of Natural Medicines*.

[43] Huang T. H.-W., Tran V. H., Duke R. K. (2006). Harpagoside suppresses lipopolysaccharide-induced iNOS and COX-2 expression through inhibition of NF-*κ*B activation. *Journal of Ethnopharmacology*.

[44] Kundu J. K., Mossanda K. S., Na H.-K., Surh Y.-J. (2005). Inhibitory effects of the extracts of Sutherlandia frutescens (L.) R. Br. and *Harpagophytum procumbens* DC. on phorbol ester-induced COX-2 expression in mouse skin: AP-1 and CREB as potential upstream targets. *Cancer Letters*.

[45] Haque A., Koide N., Odkhuu E. (2014). Mouse pyrin and HIN domain family member 1 (pyhin1) protein positively regulates LPS-induced IFN-*β* and NO production in macrophages. *Innate Immunity*.

[46] Hoshino K., Kaisho T., Iwabe T., Takeuchi O., Akira S. (2002). Differential involvement of IFN‐*β* in Toll‐like receptor‐stimulated dendritic cell activation. *International Immunology*.

[47] Kim J.-H., Kim S.-J., Lee I.-S. (2009). Bacterial endotoxin induces the release of high mobility group box 1 via the IFN-*β* signaling pathway. *The Journal of Immunology*.

[48] Toshchakov V., Jones B. W., Perera P.-Y. (2002). TLR4, but not TLR2, mediates IFN-*β–*induced STAT1*α*/*β*-dependent gene expression in macrophages. *Nature Immunology*.

[49] Koeberle A., Werz O. (2014). Multi-target approach for natural products in inflammation. *Drug Discovery Today*.

[50] Lee J., Lee I. H., Lee J. W., Kim E.-J., Kim M.-J. (2015). Study on single-dose intramuscular toxicity of Shinbaro pharmacopuncture in Sprague-Dawley (SD) rats and beagle dogs. *Journal of Korean Medicine Rehabilitation*.

[51] Lee J., Ha I. H., Kim M. R. (2015). Multiple-dose intramuscular toxicity study of Shinbaro pharmacopuncture in Sprague-Dawley rats over a 4-week period. *Journal of Acupuncture Research*.

